The article "Evaluation of Serum and Gene Expression of Galectin-4, Interleukin-27, and Complement-7 in Hepatitis C Virus-Infected Egyptian Patients" was published in 2020. Journal: Biomed Res Int.

# Evaluation of Serum and Gene Expression of Galectin-4, Interleukin-27, and Complement-7 in Hepatitis C Virus-Infected Egyptian Patients

**DOI:** 10.1155/2020/8879758

**Published:** 2020-12-15

**Authors:** Marwa S. Abdel-Tawab, Hanan H. Fouad, Dalia A. Omran, Aml E. Abdou, Shaimaa Mohamed Zaied, Alaa A. Mohamed

**Affiliations:** ^1^Medical Biochemistry Department, Faculty of Medicine, Beni-Suef University, Egypt; ^2^Medical Biochemistry Department, Faculty of Medicine, Cairo University, Egypt; ^3^Endemic Medicine and Hepatology Department, Faculty of Medicine, Cairo University, Egypt; ^4^Microbiology and Immunology Department, Faculty of Medicine, Al-Azhar University, Egypt; ^5^Clinical and Chemical Pathology Department, Faculty of Medicine, Beni-Suef University, Egypt; ^6^Medical Biochemistry Division, Pathology Department, Faculty of Medicine, Jouf University, Sakaka, Saudi Arabia

## Abstract

**Background:**

Hepatitis C virus (HCV) is considered a major global public health problem. Recently, there are great advances in HCV therapy, but there are some limitations that are creating an urgent need for assessment of some cytokines that have a potent antiviral effect in the immune system and anti-inflammatory effects to provide a potential novel immunotherapeutic target in HCV infection.

**Objective:**

This study was directed to assess the serum levels and gene expression levels of Galectin-4 (LEG4), Interleukin-27 (IL-27), and Complement-7 (C-7) and their correlation with the viral load in HCV infection. *Subjects and Methods*. This work was conducted on 80 subjects, Group 1 (*n* = 40) early detected HCV patients and Group 2 (*n* = 40) healthy controls. LEG4, IL-27, and C-7 were assessed at the protein levels by ELISA, and their gene expression was assessed by RT-qPCR. The viral load was measured by PCR.

**Results:**

There were significant elevations in the mean levels of gene expression and serum levels of all studied parameters LEG4, IL-27, and C-7 in the HCV group compared to the control group. Significant negative correlations between the viral load and each of the serum proteins and gene expressions of both LEG4 and IL-27 in HCV patients were found. The gene expression levels of LEG4, IL-27, and C-7 were positively correlated with their corresponding serum proteins in HCV patients.

**Conclusion:**

LEG4 and IL-27 showed significant negative correlations with the viral load, which could be an immune response to the control of the extent of hepatic inflammation, thus creating a potential novel immunotherapeutic approach in HCV infection for further studies or therapeutic clinical trials.

## 1. Introduction

Infection with hepatitis C virus (HCV) is a universal common disease impacting more than 177.5 million adult persons all over the world [1]. The anti-HCV seroprevalence in Egypt was 14.8% [2]. Also, there is a prevalence of occult hepatitis C virus among hemodialysis Egyptian patients who seemed to be free of HCV (negative for serum HCV tests) but have viable HCV in their tissue cells flaring up the spread of HCV from apparently uninfected persons [3]. Infection with HCV usually progresses to liver cirrhosis and hepatocellular carcinoma (HCC) with lag treatment. Because of previous bad outcomes of HCV, there is an urgent requirement for potent and early antiviral agents to stop its bad prognosis [4]. According to the balance between immunity and viremia, the good or bad prognosis is [4, 5].

Galectins are universal glycan-binding proteins or lectins that identify a lot of *N*-acetyllactosamine residues on glycoconjugates of the cell surface. Fifteen galectins have been described in mammals until now [6]. Some galectins participate at various levels in antiviral defense, from the initial recognition and blocking of the envelope and fusion glycoproteins to the activation and amplification of the innate and adaptive immune responses [7]. Some galectins were suggested to be used as viral therapeutic targets or antagonists [8].

Galectin-4 (LEG4) has two carbohydrate recognition domains (CRDs) joined by a linker peptide. In healthy people, it is mainly expressed in the gastrointestinal tract. It was reported that LEG4 had a dual role in control [9] and promotion of intestinal inflammation [10]. Moreover, high levels of it were observed in hepatitis B virus (HBV) patients, suggesting its control role in liver inflammation [11]. Furthermore, it is upregulated in HCC [11], and gastric cancer [12] was reported. However, there were controversial studies about its expression in cancers that revealed its downregulation in human colorectal cancer [13], suggesting its tumor suppressor effect [13].

Immunoregulatory cytokines affect the progression of HCV chronic infection and the magnitude of liver damage. From these cytokines, interleukin-1 (IL-1) correlates with the severity of HCV disease [14]. Also, there is an association between the IL-12 B gene polymorphism and the staging of HCV disease [15].

Interleukin-27 (IL-27) is one of the IL-6/IL-12 family of cytokines released by activated antigen-presenting cells. IL-27 was reported to have antiviral and anti-inflammatory effects in viral infection [16].

Failure of the old therapeutic protocol of IFN-alpha therapy is accompanied by upregulation of some genes as a compensatory mechanism; IL-27 was reported to be one of these genes suggesting the synergistic relation between IL-27 and IFN-alpha in vitro [17]. All previous data need more studies to evaluate the role of IL-27 in viral hepatitis.

The complement system (CS) has a vital role in the interaction between innate and adaptive immunity [18]. There are more than fifty proteins on the cell plasma membranes that belong to CS, which are assembled in three pathways: classical, lectin, and alternative pathways which are independent but interactive pathways [18].

The liver synthesizes most CS proteins except some proteins like Complement-7 (C-7), which is formed in monocytes and macrophages. C-7 has a vital role in the membrane attack complex (MAC) formation [19] which is formed on the cell membranes at the terminal phase of CS activation and has a role in the cell lysis [19].

C-7 inherited deficiency or polymorphism is associated with bacterial infection [20], and inflammatory diseases are associated with fibrosis like HCV infection; low C-7 leads to evading hepatic apoptosis with consequent HCV disease progression and tumor development due to low activation of MAC [21].

C-7 was suggested to be a potential tumor suppressor [22]. Although C-7 has a role in limiting virus replication and inflammation with enhancing tissue regeneration, it may be involved in fibrogenesis and cancer [23].

Following on from previous studies, the present study was conducted to evaluate the serum levels and gene expression levels of LEG4, IL-27, and C-7 and to assess the correlation between them and the viral load in HCV-infected Egyptians. Few studies evaluated them in HCC [11, 21, 24], but no studies evaluated LEG4 and C-7 in HCV infection. So, up to our knowledge, this is the first study evaluating the serum levels and gene expression levels of LEG4 and Complement-7 (C-7) in HCV infection. Assessment of the protein and gene expression levels was implemented by ELISA and RT-qPCR, respectively.

## 2. Patients and Methods

The present study was conducted on 80 subjects, Group 1 (*n* = 40) HCV patients and Group 2 (*n* = 40) healthy controls. HCV mRNA was assayed by quantitative PCR. Patients were selected from the Gastroenterology and Hepatology Department of Kasr-Alainy Hospital and outpatient clinic during the period from January to April 2018. The study was carried out in compliance with the guidelines and principles of the Helsinki Declaration [25]. Written consent forms were taken from all patients before enrollment in the study. The exclusion criteria include psychiatric, neurological, or any other disorder that prevented informed consent, presence of any other type of malignancy, patients starting chemotherapy or radiotherapy, and HBV or HIV coinfection. The laboratory investigations were conducted in the Biochemistry & Molecular Biology Unit, Faculty of Medicine, Cairo University.

### 2.1. Assay of HCV mRNA

According to Rolfe et al. [26], HCV mRNA was detected by quantitative PCR using a Human artus HCV RG RT-PCR Kit (Qiagen, Germany, Cat No./ID: 4518263).

### 2.2. Assay of Serum Protein Levels of LEG4, IL-27, and C-7

The three studied parameters were assessed in the serum using the commercial ELISA kits according to the manufacturer's recommendations: Human LEG4 ELISA Kit (ab213785), Human IL-27 ELISA Kit (ab83695), and Human Complement-7 ELISA Kit (ab125964) supplied by Abcam (USA).

### 2.3. Assay of Gene Expression Levels of LEG4, IL-27, and C-7

Gene expression levels of the three parameters were conducted by real-time PCR using the StepOnePlus™ real-time PCR system (Applied Biosystems, USA). Total RNA was extracted from the whole blood using the QIAamp RNA Blood Mini Kit (Qiagen, USA, Cat No./ID: 52304). The extracted RNA was quantified by spectrophotometry (Jenway, USA) at 260 nm.

### 2.4. Primer Sequence

PCR primers are shown in Table 1 and are taken from GenBank RNA sequences cited at http://www.ncbi.nlm.nih.gov/tools/primer-blast. The ideal primer pair was selected with optimal factors including melting temperature (Tm: 60 to 65°C) and applicant length of about 90 to 200 bp.

### 2.5. Reverse Transcription Quantitative PCR Using SYBR Green

The StepOnePlus™ real-time PCR system was used in the analysis using software version 3.1 (Applied Biosystems, USA). Optimization of the annealing temperature was conducted for the PCR protocol and for the primer sets.

All cDNAs were prepared for all gene markers, glyceraldehyde 3-phosphate dehydrogenase (GAPDH), and nontemplate negative control. Five microliters of total RNA was used to generate cDNA using 20 pmol antisense primer and 0.8 *μ*L AMV reverse transcriptase at 37°C for 60 min. The relative abundance of mRNA species was evaluated using the SYBR® Green method (Applied Biosystems, CA, USA). The annealing temperature of 60°C was optimized for all primer sets. Real-time polymerase reaction was performed in 25 *μ*L reaction volumes consisting of SYBR Green Master Mix, 3 *μ*L of cDNA, and 900 nmol/L of every primer. Amplification conditions were conducted according to the manufacturer's specifications: 2 min at 50°C, 10 min at 95°C, 40 repeated cycles with 15 s denaturation, and 10 min of annealing/extension at 60°C.

### 2.6. Calculation of Relative Quantification (Relative Expression)

The relative gene expressions of all assessed genes were calculated using the comparative cycle threshold (Ct) method. The PCR data results show the Ct values of the target genes and the housekeeping gene (GAPDH). A negative control sample was that no template cDNA was used. The data were calculated using the Applied Biosystems StepOnePlus™ software. All values were normalized to the housekeeping gene GAPDH and expressed as fold changes relative to the background levels found in the control samples. Relative quantitation of target gene expression (RQ) was calculated according to the following equations [27]:

(1) $$\begin{array}{c} \Delta \text{Ct}=\text{Ct assessed gene}-\text{Ct reference gene},\\ \Delta \Delta \text{Ct}=\Delta \text{Ct sample}-\Delta \text{Ct control gene},\\ \text{RQ}=2^{-\left(\Delta \Delta Ct\right)}. \end{array}$$

### 2.7. Statistical Analysis

Statistical Package for the Social Sciences (SPSS) version 16.0.1 (SPSS Inc., Chicago, IL, USA) was utilized. The data were described as mean ± SD. The differences between groups were analyzed by the Kruskal-Wallis test, Shapiro-Wilk test, and *t*-test. Post hoc testing was performed by the Tukey test to compare the difference among the groups. Simple linear correlation (Pearson's correlation coefficient test) (*r*) was also done to test for linear relations between the studied genes and clinical variables. *p* value is considered significant if *p* < 0.05.

## 3. Results

The clinical data of the studied groups are shown in Table 2 with high significant differences (*p* < 0.001) in the mean levels of platelets, hemoglobin (HB), international normalized ratio (INR) (blood clotting time), alanine aminotransferase (ALT), aspartate aminotransferase (AST), alkaline phosphatase, and albumin in the HCV group compared to the control group. Moreover, the mean levels of the viral load in the HCV group are shown in Table 2.

There were high significant elevations (*p* < 0.001) in LEG4 gene expression, LEG4 serum protein, IL-27 gene expression, IL-27 serum protein, and C-7 serum protein in the HCV group (5.69 ± 2.35, 479 ± 201, 0.53 ± 0.15, 1.85 ± 0.63, and 7.05 ± 1.2, respectively) compared to the control group (0.45 ± 0.12, 37.75 ± 10.24, 0.53 ± 0.15, 1.5 ± 0.40, and 5.8 ± 0.85, respectively) as shown in Figures 1–3. Also, there was a significant elevation (*p* < 0.05) in C-7 gene expression in the HCV group (1.1 ± 0.19) compared to the control group (0.9 ± 0.15) as shown in Figure 3.

Significant negative correlations were found between LEG4 serum protein (*r* = −0.845, *p* < 0.001) and LEG4 gene expression levels (*r* = −0.852, *p* < 0.001) and IL-27 protein (*r* = −0.779, *p* < 0.001) and IL-27 gene expression levels (*r* = −0.367, *p* = 0.02) with the viral load in the HCV group as shown in Figures 4 and 5 while there were no significant correlations were found between the gene expression and serum protein levels of C-7 with the viral load in the HCV group.

The gene expression levels of LEG4, IL-27, and C-7 were positively correlated with LEG4 serum protein levels (*r* = 0.999, *p* < 0.0001), IL-27 serum protein levels (*r* = 0.981, *p* < 0.001), and C-7 serum protein levels (*r* = 0.984, *p* < 0.001), respectively, in the HCV group as shown in Figure 6. All studied parameters were expressed as ng\mL.

## 4. Discussion

HCV disease is considered a major global public health problem. There are great advances in HCV therapy. Using the old therapeutic protocol of ribavirin, peg-IFN-alpha showed that more than half of treated patients were unable to clear the virus constantly or to avoid the long-term complications of chronic viral infection [28]. Moreover, the recent protocol of direct-acting antivirals (DAAs) may be associated with drug resistance due to the high mutation rate of the HCV RNA polymerase [29]. Therefore, evaluation of some cytokines that have a potent antiviral effect in the immune system and anti-inflammatory effects may provide a potential novel therapeutic approach in HCV infection.

The present study was conducted to assess the serum levels and gene expression levels of LEG4, IL-27, and C-7 and their correlation with the viral load in HCV patients.

The current work showed high significant elevations in the mean levels of gene expression and serum protein levels of LEG4 in the HCV group compared to the control group. These results might be explained as a response to liver inflammation due to the anti-inflammatory properties of LEG4, which were reported in intestinal inflammatory diseases through either interacting with activated T cells via CD3 binding and enhancing T cell apoptosis or decreasing proinflammatory cytokine synthesis [9]. To assume if LEG4 use exerts similar anti-inflammatory mechanisms in liver inflammation needs further studies.

Moreover, a high significant negative correlation between the mean levels of gene expression and serum protein levels of LEG4 with the viral load was found in the HCV group. This finding suggested an antiviral effect of LEG4 in HCV like other galectins which were reported to be upregulated in some viral infections, suggesting their antiviral defense through activation and augmentation of immune responses [7, 8].

It has been reported that Galectin-3 had antiviral effects in HCV infection through different mechanisms. Galectin-3 restricted the proinflammatory response with IL-6 in HCV, decreasing chronic inflammation [30]. Moreover, Galectin-3 was used as a prognostic marker of cirrhosis in HCV disease [31].

On the contrary, Galectin-9 was reported to establish and maintain chronic hepatitis C viral infection. Galectin-9 had a role in the inhibition of adaptive immunity in HCV disease through the induction of HCV-specific T cell apoptosis and the increase of inhibitory Treg cells [32, 33].

The present study suggested an antiviral effect of LEG4 in HCV infection, but further studies are needed to explore the mechanisms involved in its antiviral effect in HCV disease.

Cai et al. [11] reported similar results but in patients with HBV infection. They explained their results as an immune response against liver inflammation via the induction of T cell apoptosis by LEG4 by decreasing proinflammatory cytokine secretion [9]. Similarly, Kondoh et al. [34] showed that LEG4 gene expression was increased in liver tissues of cirrhotic HCV patients compared to the control group but was still decreased compared to the HCC group.

The current study showed high significant elevations in the mean levels of gene expression and serum protein levels of IL-27 in the HCV group compared to the control group.

Moreover, a high significant negative correlation between the mean levels of both the gene expression and serum protein levels of IL-27 with the viral load was found in the HCV group.

These findings coincided with Houssen et al. [24] who showed elevated serum IL-27 in the HCV group compared to the control group with a significant negative correlation between the serum levels of IL-27 and the serum viral load in HCV patients. They assumed that their results were due to the antiviral activity of IL-27, as it was known that IL-27 could induce some antiviral STAT1-dependent genes and has a similar action to that of IFN-*α* against hepatic viral infection [35]. Wang et al. [36] showed elevated gene expression and serum protein levels of IL-27 in HBV patients which still were lower than the corresponding levels in liver cirrhosis and HCC suggesting that IL-27 might be used in the clinical management of HBV establishing novel therapeutic targets in this disease.

Similarly, Zhu et al. [37] and Cao et al. [38] reported that HBV enhances IL-27 expression, while the latter showed the synergetic mechanism between IL-27 and IFN-*λ*1 inhibiting HBV protein expression and virus replication through type I IFN.

The present findings and previous studies regarding IL-27 could be explained by the effect of IL-27 on T cells and on hepatocytes and suggested that IL-27 induced the antiviral Th1 cell synthesis; additionally, both IL-27 and interferon-*α* have a similar antiviral mechanism through induction of STAT1-dependent genes blocking the differentiation into Th17 cells and iTreg cells [39].

IL-27 strongly induced STAT1-dependent pathways and weakly induced STAT3-dependent pathways implicated in flaring up the viral infection and HCC progression in liver viral infection, suggesting the probable use of IL-27 as a safe treatment in viral hepatitis [40, 41]. Further studies are recommended to assess IL-27 effects on viral replication, its expression in chronic viral infection, and its effect on the outcome of the disease.

The current work showed significant elevations in the mean levels of gene expression and serum protein levels of C-7 in the HCV group compared to the control group. These results could suggest an immune response as C-7 is a key element of the lytic pathway of the complement system, resulting in membrane attack complex (MAC) establishment controlling the exaggerated proinflammatory response [19] abolishing the infected hepatocytes by adaptive immunity, but it was reported to be involved in fibrogenesis [42].

The current work showed no significant correlation between the viral load and each of the mean levels of C-7 serum protein and its gene expression. These results might be explained by HCV utilization of various mechanisms to evade the complement-mediated lytic pathway. HCV was reported to regulate the complement synthesis and hinder the MAC formation. Although HCV forcibly stimulates the complement cascades, it is not eliminated by the complement system but often progresses into a chronic disease in most cases [43, 44].

Mas et al. [45] coincided with the present study as they showed overexpression of 18 proteins in the HCV group than the control group in cirrhotic HCV patients awaiting liver transplantation. LEG4, IL-27, and C-7 were some of these proteins.

The present results showed high significant positive correlations between the gene expression and serum protein levels of each studied parameter. These results were logical as the serum proteins were increased secondary to the upregulation of their genes.

## 5. Novelties

Novelties of the study are as follows:

- Assessment of both genes and their corresponding proteins with correlations between genes and proteins to validate our results
- Correlations between the viral load and all of the studied parameters
- Recommendations of immunotherapy regarding LEG4 and IL-27 in HCV infections

## 6. Limitations

Limitations of the study are as follows:

- Conducting the study on another patient group who received a direct antiviral therapeutic regimen to evaluate the effect of treatment on the studied parameters
- Conducting the study on different governorates, i.e., multicenter study

## 7. Conclusion

There were significant elevations of LEG4, IL-27, and C-7 levels in HCV-infected patients. Moreover, LEG4 and IL-27 showed a significant negative correlation with the viral load, suggesting their antiviral and anti-inflammatory effects to control the extent of hepatic inflammation, thus creating a potential novel immunotherapeutic approach in HCV infection which needs further studies and therapeutic clinical trials.

## Figures and Tables

**Figure 1:** Mean ± 1 SD Galectin-4 protein and gene expression in studied groups. ^∗∗^Statistically high significant differences compared to the corresponding values in the control group (*p* < 0.001).

**Figure 2:** Mean ± 1 SD IL-27 protein and gene expression in studied groups. ^∗∗^Statistically high significant differences compared to the corresponding values in the control group (*p* < 0.001).

**Figure 3:** Mean ± 1 SD C-7 protein and gene expression in studied groups. ^∗∗^Statistically high significant differences compared to the corresponding values in the control group (*p* < 0.001). ^∗^Statistically significant differences compared to the corresponding values in the control group (*p* < 0.05).

**Figure 4:** Correlations between the Galectin-4 protein (*r* = −0.845, *p* < 0.001) and Galectin-4 gene expression levels (*r* = −0.852, *p* < 0.001) with the viral load.

**Figure 5:** Correlations between the IL-27 protein (*r* = −0.779, *p* < 0.001) and IL-27 gene expression levels (*r* = −0.367, *p* = 0.02) with the viral load.

**Figure 6:** Correlations between the gene expression and serum protein levels of each studied parameters in the HCV group: Galectin-4 (*r* = 0.999, *p* < 0.0001), IL-27 (*r* = 0.981, *p* < 0.001), and C-7 (*r* = 0.984, *p* < 0.001).

**Table 1:** PCR primers.

Gene	Sequence	Gene bank accession number
Galectin-4 (LEG4)	F: 5′-CTCAGACGTCGCCTTCCACT-3′ R: 5′-GGCTGTTCAGCTGTTGATGG-3′	NM_006149.4
Interleukin-27 (IL-27)	F: 5′-GACGGCAGGCGACCTTG-3′ R: 5′-GCTGACTGTGAACTCCCTCC-3′	NM_145659.3
Complement C-7 (C-7)	F: 5′-GACCCCCGGAACTTTGGATT-3′ R: 5′-TTAGCCATGATCTGCCCAGC-3′	NM_000587.4
GAPDH	F: 5′-GATGCTGGTGCTGAGTATGTCG-3′ R: 5′-GTGGTGCAGGATGCATTGCTGA-3′	XR: 598347.1

PCR: polymerase chain reaction; NM: neutrophil migration (genetic locus); GAPDH: glyceraldehyde 3-phosphate dehydrogenase; F: forward primer; R: reverse primer.

**Table 2:** Clinical data of the studied groups.

	HCV group (*M* ± SD) *n* = 40	Control group (*M* ± SD) *n* = 40
WBCs (cells/microliter)	5.81 ± 2.67	5.1 ± 2.22
Platelet (10^3^ cells/microliter)	128.09 ± 91.88^∗∗^	243 ± 88.4
HB (g/dL)	10.22 ± 2.42^∗∗^	13.54 ± 2.76
INR	1.59 ± 0.39^∗∗^	1.0 ± 0.02
ALT (*μ*/L)	46.53 ± 23.05^∗∗^	22.64 ± 6.2
AST (*μ*/L)	77.22 ± 39.04^∗∗^	21.32 ± 6.5
Alkaline phosphatase (*μ*/L)	136.84 ± 76.12^∗∗^	73.54 ± 15.32
Albumin (g/dL)	2.84 ± 0.73^∗∗^	3.95 ± 0.4
Bilirubin (mg/dL)	1.45 ± 1.90^∗∗^	0.7 ± 0.28
Viral load (×10^5^ IU/mL)	5.43 ± 1.87	—

Values are presented as *M* ± SD (mean ± standard deviation). HCV: hepatitis C virus; *n*: number of cases; WBCs: white blood cells; HB: hemoglobin; INR: international normalized ratio (for blood clotting time); ALT: alanine aminotransferase; AST: aspartate aminotransferase. ^∗∗^Statistically high significant differences compared to the corresponding values in the control group (*p* < 0.001).

## Data Availability

Readers can access the data supporting the conclusions of the study by requesting them from the authors.

## Abbreviations

HCV: Hepatitis C virus
HCC: Hepatocellular carcinoma
LEG4: Galectin-4
IL-27: Interleukin-27
C-7: Complement-7.
